RETRACTED

# Novel insights on different treatment of magnesium alloys: A critical review

**DOI:** 10.1016/j.heliyon.2022.e11712

**Published:** 2022-11-17

**Authors:** B. Elambharathi, S. Dharani Kumar, V.U. Dhanoop, S. Dinakar, S. Rajumar, Shubham Sharma, Vineet Kumar, Changhe Li, Elsayed Mohamed Tag Eldin, Szymon Wojciechowski

**Affiliations:** a Department of Mechanical Engineering, KPR Institute of Engineering and Technology, Coimbatore, India; b Department of Mechanical Engineering, Institute of Technology, Hawassa University, Ethiopia; c School of Mechanical and Automotive Engineering, Qingdao University of Technology, Qingdao, 266520, China; d Mechanical Engineering Department, University Center for Research and Development, Chandigarh University, Mohali, 140413, Punjab, India; e Department of Automobile Engineering, Chandigarh University, Mohali, 140413, Punjab, India; f Future University in Egypt, New Cairo, 11835, Egypt; g Poznan University of Technology, Poznan, 60-965, Poland

**Keywords:** Magnesium alloys, Heat treatment, Tensile strength, Corrosion resistance, Microstructure

## Abstract

Magnesium alloys are extensively used for weight reduction in automotive and aircraft applications. This research presents the effect of heat and cryogenic treatment on aluminium-zinc-based Mg alloys. Both treatments can improve the mechanical and corrosion properties of the AZ series Mg alloy. The review deals with a broad understanding of the microstructure changes that occur during heat and cryogenic treatment of Mg alloy. The mechanical and corrosion characteristics of heat and cryogenic treated AZ31, AZ91, AZ63, and AZ80 Mg alloys are discussed. The essential strengthening mechanisms of heat and cryogenic treated AZ series Mg are discussed with microstructure changes. This review has also shown a few gaps in research on the selection of suitable pre- and post-treatment processes for Mg alloy. The effects on grain refinement and the formation of secondary phase particles are discussed in detail. The related crystallographic plane, twining, and dislocation changes are out of the scope of this review. Finally, the correlations of the above changes to mechanical properties are the directions of the future.

## 1 Introduction

Alloys of magnesium have been very popular in recent years, owing to characteristics like high specific strength, lightweight, and so on. Mg alloys are the lightest alloys, making them excellent contenders for application in a variety of industries, including automotive and aerospace, as well as medical, electronic, and sporting goods. Another distinguishing aspect of magnesium is its hexagonal close-packed crystal structure, which renders it less malleable at ambient temperature. However, traditional magnesium alloys like AZ31, ZK60, and AZ61 have several drawbacks, including weak creep resistance, low tensile strength, and low corrosion resistance, which have limited their use in a variety of industries. The aerospace industry's quest for materials of lightweight that can work under high conditions of demand has traditionally spurred magnesium alloy research. Designers have always been drawn to magnesium alloys because of low in their density. This is a big reason why wrought products and magnesium alloy castings are so popular. There has been high demand in recent years for better corrosion resistance, and new magnesium alloys have shown substantial gains in this area. Due to enhancements in characteristics of mechanical and resistance to corrosion, magnesium alloys are becoming more popular for aerospace and other specialised applications. Figure 1 shows the application of magnesium alloy.

RETRACTED

**Figure 1:** Applications of Mg alloy.

Magnesium is employed in a broad range of applications, including metallurgical and medical applications, as well as pyrotechnic and chemical applications. Magnesium alloys' high strength-to-weight ratio is frequently cited as a primary rationale for using them in engineering designs. Magnesium alloys have desirable features such as cast ability, machinability, high stiffness-to-weight, and superior damping, which all play a role in the material selection process. Industrial, automotive, commercial, materials handling, and aerospace equipment are all structural uses. Magnesium alloys are used in industrial machinery, such as printing machines and textiles. Brake pedal support brackets and clutch, manual transmission housings, and steering column lock housings are among the automobile applications. Gravity conveyors, grain shovels, and dock boards are examples of materials-handling equipment. Computer housings, baggage, handheld tools, and ladders are examples of commercial applications. Because magnesium alloys are lightweight and display good stiffness and strength at both room and increased temperatures, they are ideal for aerospace applications.

The present review paper mainly concentrated on the effect of heat and cryogenic treatment of AZ series Mg alloy. The microstructure changes before and after treatments have correlated with mechanical and corrosion properties is discussed. This review also provides a clear idea about the selection of suitable treatment processes for improving the properties of AZ series Mg alloy.

## 2 Methods for improving mechanical properties of AZ Mg series alloys

### 2.1 Heat treatment

In Mg alloys, because of their adaptability to be in a variety of forms such as tubes, sheets, rods and so on, one-step high-ratio extrusion is used. It has been proven that a single pass of strong deformation produces fine grains and higher-angle grain boundaries than numerous runs of high accumulated strain. The effect of the extrusion ratio on elongation was found to be greater than that on elongation, and tensile strength improved as the extrusion ratio was increased. After homogenization for 2 h at 300 °C and for 5 h at 400 °C [1], the as-cast AZ61 alloy was extruded at an extrusion ratio of 166:1 to produce a sheet [1]. The homogenised alloy at 390 °C was extruded with a 2.1 m min^−1^ extrusion flow rate [1]. During the extrusion process, a thermocouple was placed within the die to calculate the relative temperature of the shear zone. The temperature was raised to 420 °C [1] due to friction and plastic deformation during the extrusion operation. Following this, the sheet was aged at 170 °C in a furnace before being air-cooled naturally [1]. Vickers microhardness testing under a load of 50 g for 15 s was used to analyse the ageing response in mechanically polished samples [1].

RETRACTED

### 2.2 Equal channel angular pressing

ECAP is best suited for use in industrial applications since it uses repeated extrusion processes to create a significant shear strain. It may be used on a wide range of alloys and metals to produce fine grains with excellent physical and mechanical qualities. The creation of mechanisms and the fine grains driving the strength to high levels seen are two essential components of SPD techniques that have recently attracted a lot of attention in the literature. The most commonly used materials in SPD-ECAP research are aluminium and its alloys, copper, and titanium, with titanium being seriously examined for orthopaedic implants. By forcing the workpiece along with a die of the same cross-sectional form as two channels, considerable shear strain is introduced in the work piece. The cross-sections of both channels are similar; the product can again be fixed into the channel and forced along with the die. Fine grains are produced via extrusion via ECAP die by accumulating enough strain to break down the microstructure. On the hydraulic press, components were at 200 °C (473 K) [2] under ECAP. A deformation path was used (90° rotation along the longitudinal axis in the same direction). The ECAP procedure involves extruding the component along with an L-shaped internal channel tool [2] without changing the sample's cross-section. The sample is placed in the channel, which is vertical from above, and then extruded with the help of the tool. The technique is continued until the material has undergone the desired degree of distortion, resulting in the refinement of the structure. For the ECAP process, different types of deformation pathway alterations are conceivable. ECAP was done using a die that changed the tool shape. The process efficiency was enhanced by combining ECAP with Twist Extrusion [2]. That tool has a built-in helix with a 30° spiral angle [2]. The ECAP tool is made of HOTVAR, a material that has improved strength stability at higher temperatures during forming processes.

RETRACTED

### 2.3 Hydrogenation disproportionation desorption recombination treatment

Ultrasonic washing in acetone was used to remove the oxide scale with the help of Sic paper from the alloy plate's surface [3]. Following that, the powders were given the hydrogenation disproportionation desorption recombination treatment process. Under 7 MPa hydrogen pressure, the components were heated to 350 °C [3] for the hydrogenation stage, then kept at this temperature for 24 h. The evacuation treatment was carried out for the stage of dehydrogenation using a rotary oil pump for 3 h [3] at the same temperature range.

## 3 Results and discussions

### 3.1 Microstructure changes in AZ31 alloy

The coarse, inhomogeneous distribution of β-Mg_17_Al_12_ throughout the grain boundaries is visible [4] in the microstructure of AZ31's base material. The microstructure of the specimens changed significantly after heat treatment and FSP. The typical microstructure of AZ31 alloy after FSP and heat treatment was homogenous and recrystallized grains [4]. The nugget zone exhibits a fine grain structure when compared to the surrounding thermo mechanically damaged zone [5]. XRD analysis was used to identify the phases present in the base material. After the FSP double pass [5], which was followed by thermal processing], the phase peaks were lowered to considerable extent. Figure 2(a, b) shows the AZ31B Mg alloy before and after heat treatment. As evidenced by this the phase is finely dispersed across the agitated zone. The microstructure of the AZ31 magnesium alloy changes after heat treatment. It's clear that there are twins present. At the same time, as the temperature drops to 77 K [6], the amount of twinning increases. This magnesium alloy, which is treated via high-pressure torsion, is a good alternative for making an ultra-fine-grained AZ31 alloy.

**Figure 2:** Microstrcutre of Cast AZ31B Mg alloy (a) before heat treatment (b) after heat treatment.

The formation of small particles was seen in the heat treated samples. However, it confirmed by the microstructure image. By HPT under a 6.0 Gpa [7] applied pressure at ambient temperature an annealed alloy with an initial coarse grain size of 35 μm [7]. It is difficult to process when subjected to ECAP because of challenges obtaining consistent refinement of grain and the potential of forming cracks inside billets.

RETRACTED

### 3.2 Microstructure of AZ61 Mg alloy

At normal temperatures, the microstructure of the AZ61 magnesium alloy reveals larger granules [8]. In the magnesium alloy matrix, spheroidized particles and discontinuous precipitates are dispersed. The grains were loosely oriented after heat treatment, and the hardness was significantly reduced [8] due to atom vacancy. After severe cryogenic treatment, aluminium's solubility in magnesium decreases, and the β-phase forms along lines of dislocation and boundaries of grain [9]. This steadily grows throughout the therapy and does not disappear after the recovery of the temperature process. During the deep cryogenic treatment, stresses in internal and corresponding strains are formed, causing dislocation propagation and the formation of β-phase [9] and sub crystals. Grain refinement is caused by these microstructural changes [10]. Because of the kinetic energy of the atoms and severely low temperatures, proliferation is difficult, which slows the expansion of the β-phase [10]. This results in the creation of a network of phases continuously with very tiny particle sizes [9]. The welded metal structure is a non-equilibrium crystal product due to the enormous input of heat during the process of welding and quick cooling following the process of welding. As a result, the zone of weld has a different phase composition than the base metal. The grain sizes in the weld zone are the smallest, and the area of the grain boundary is larger than the zones in other areas. When the deep cryogenic treatment period was extended to 4 h, the phase of the zone in the weld improved dramatically [9]. The joint area of the base material increased when the temperature of cryogenic treatment was reduced, notably in the heat-affected zone, where sub grain formation was simpler. Figure 3(a, b) depicts the microstructure of before and after cryogenic treatment. Cryogenic treatment significantly increased the formation of Mg_17_Al_12_ precipitate particles.

**Figure 3:** Microstrcture (a) before cryogenic treatement (b) after crygenic treatment.

When it comes to the microstructure of AZ61 magnesium alloy, α-Mg is the matrix, and the secondary phase is a substantial quantity of β-Mg_17_Al_12_ [11]. The cast material was treated at 410 °C [12] for homogenization for 24 h. Secondary beta particles dissolve in the matrix, leaving a trace on the grain boundary [12] and improving the material's ductility. As a result, adding Sic particles to a magnesium alloy matrix composite has a considerable impact on grain refinement. When 1 wt% SiCp is added to pure AZ61 alloy, the average grain size drops, but when 2wt% SiCp is added, the average grain size increases [12] when compared to 1wt%. Because of the right selection of stirring parameters such as stirring speed, stirring time, and so on, the microstructure composites SiCp must be mostly diffused throughout the matrix. During the tensile test, the uniformly dispersed SiCp enhanced the dislocation density, which boosted the material's strength. During one pass of the equal channel angular pressing operation on AZ61 magnesium alloy, there is a high dislocation density, the creation of shear bands, and the grains [2] have a somewhat elongated shape. The microstructure is refined and the grain size is reduced [2]. Because the operation was carried out at 200 °C [2], the reduced dislocation density suggests that dynamic recrystallization happened.

RETRACTED

### 3.3 Microstructure of AZ63 Mg alloy

The microstructure of the AZ63 Mg die-cast alloy shows grains of primary phase and β- Mg_17_Al_12_ phase heterogeneously dispersed in the matrix. After cooling to room temperature after 16 h of solution heat treatment at 400 °C [13], all intermetallic phases, particularly β- Mg_17_Al_12_, vanished. It is apparent that the microstructure has changed. At 160 °C, the microstructure of the aged sample [13] is identical to that of the air-cooled sample. In other words, after aging for 1 h, very little segregation of the β- Mg_17_Al_12_ phase occurred at the grain boundaries and within the grains. Discontinuous phase precipitation often preferentially initiates part of the grain boundaries, as evidenced by the thick lamellar development of α-Mg and β- Mg_17_Al_12_ in the grains. The amount and consistency of the phase increased at the grain boundaries, within α-Mg grains as a result of regional coarse segregation at the grain boundary. It is observed that the microstructure differs from the other aged microstructures after aging time of 12 h [13]. Instead of precipitation as a lamellar structure in the grains, a thick regional precipitation of β- Mg_17_Al_12_was observed at the grain boundaries of the sample, indicating that aging for 12 h at 160 °C [13] is not sufficient to obtain a homogeneous microstructure for the obtained Mg alloy AZ63. During aging at 160 °C for 1–12 h [13] the grain boundaries of the microstructure thicken and a minuteβ- Mg_17_Al_12_ phase precipitates in the grains. If boundaries or lamellar precipitates are seen in the α-matrix in a 1hed sample, it can be concluded that there is not enough time for the β-phase to precipitate. During the aging process, the β-Mg_17_Al_12_ phase formed a lamellar eutectic structure while the α-matrix formed islands. Figure 4 shows the microstructure image of heat treated AZ63 Mg alloy. In the case of Mg–Al alloys, the lamellar phase can also be produced by cellular precipitation of the β-phase from α-grains. The lamellar eutectic phase in the structure increases with increasing aging time.

RETRACTED

**Figure 4:** Microstructure of heat treated AZ63 Mg alloy.

The microstructure of AZ63 alloy is affected by both the temperature of the mould and the amount of MgCO_3_ refiner used. As the temperature increases and the eutectic beta phase decreases, the Mg-alpha particles in the microstructure gradually coarsen, coalesce and develop into small grains [14]. Plastic deformation begins at the points of contact and the magnitude and degree of deformation increases as the temperature of the mould increases. Recrystallization is incomplete and if the alloy dissolves it can continue. High forming temperature thixoforging and solution heat treatment is a new method for producing components with small and consistent equiaxed grains. The microstructure changed as the amount of added MgCO_3_purifier increased [14] and the number of irregularly linked large particles, spherical particles and small particles decreased, as did the number of eutectic beta phases. As a result, the shape of the primary particles changes and the Al content in the liquid phase decreases. As the amount increased from 0% to 0.6% [14], the degree and degree of distortion of the alpha-Mg particles decreased and then increased. The substance of the impact can be attributed to two factors such as the change in morphology of the primary particles in the semi-solid ingot and the change in the Al content in the liquid phase. Between 0 and 0.6%, the geometry of the primary particles dominates for plastic deformation, but when the amount reaches 0.6% [14], the Al concentration of the liquid phase promotes the deformation. In all cases, as the amount increased, the Al concentration in the liquid phase decreased due to depletion by inducing the Al_4_C_3_ nucleation substrate, and thus the beta eutectic phase decreased. In addition, the particles in the dissolved microstructures became more homogeneous over time and the particle size decreased.

### 3.4 Microstructure of AZ91 Mg alloy

The as-received alloy microstructure was enhanced using cryogenic treatment and friction stir processing in the microstructure of AZ91 in the presence of alpha-Mg, β-Mg_17_Al_12_, and n-AlMn phases [15]. The cryogenic treatment of grains after the precipitation of beta-the cryogenic deep treatment, the microstructure of the as-received AZ91 alloy changed to some extent [15]. The microstructure of the beta-phase precipitates changed dramatically following DCT, and these microstructure changes polished the grains. The matrix was filled with coarsely divided eutectic beta-phase. When compared to as-received, this microstructure alteration after DCT resulted in an improvement in the alloy's mechanical properties. When compared to samples without DCT, microstructure research demonstrates that DCT causes additional linkage [15] as well as a change in grain orientation. According to several experts, the microstructure of AZ91 is mostly made up of alpha-Mg and beta-Mg_17_Al_12_ phases. The AZ91 alloy contained alpha-Mg, beta-Mg_17_Al_12_, and n-AlMn phases. The island-like second phases of Mg_17_Al_12_ at the boundaries of grain are surrounded by lamellar Mg_17_Al_12_ in the microstructure of as-cast AZ91. Mg_17_Al_12_ point-like precipitates are distributed uniformly at the boundaries of the grain [16] after semi-solid squeeze casting. The Mg_17_Al_12_ phases at the boundaries of the grain are dissolved in the matrix of Mg after T4 treatment, and secondarily precipitate into the grain interior from near the grain boundaries. After T6 heat treatment, the average size of the grain is 17.01 μm [16], the size of the second phase is 0.50 μm, and the volume fraction of the second phase is 23.05 wt.% [16] when the squeezing temperature is 575 °C [16].

RETRACTED

The major matrix phase of alpha Mg is present in the alloy that is cast into a step-like mould. Berry is formed in the main matrix by eutectic and intermetallic phases spreading along grain boundaries [17]. These phases are thought to be eutectic Mg–Al and intermetallic Mg_17_Al_12_ are shown in Figure 5.

**Figure 5:** Microstructure of heat treated cast AZ91 Mg alloy.

As the cooling rate increased, the alloy's grain structure deteriorated [17] and the intermetallic phases generated at the grain boundaries fragmented. Rapid cooling also modified the phases of the grain boundaries of the AZ91 alloy. The Mg_2_Si intermetallic phase formed at normal temperature with the addition of Si, and the Mg_2_Si phase fragmented the Mg_17_Al_12_ phase. The shape of the Mg_2_Si phase is also observed to change as the cooling rate increases [17]. The addition of Ti reduces the as-cast alloy grain size [18] while also forming metallic compounds that can enhance the fraction of alpha magnesium phases while decreasing the amount of beta Mg_17_Al_12_ phases.

### 3.5 Microstructure of AZ80 Mg alloy

The initial extruded fine grains in AZ80 after T4 heat treatment grew consistently (30 m) and developed into equiaxed grain morphologies. The banded eutectic β-phases, and also small eutectic β-phase particles, were dissolved into the matrix. However, there is still a trace amount of bulk Al_8_Mn_5_ intermetallic complexes at the grain boundaries. As a result, the T4 treatment did not involve the Al_8_Mn_5_ intermetallic complex with a high melting point. The banded eutectic β-phases are still visible after T5 (15 h at 200 °C) treatment [19], but in a considerable amount, the precipitation band was formed as a result of newly generated β-phases precipitating around the eutectic β-phases. This implies that the eutectic β-phase locations had a significantly higher Al content than in the other matrix regions, which favoured β-phase precipitation. In general, lamellar-shaped discontinuous precipitate (DP) tends to form at high-Al grain borders and extends inside the grains [19]. The precipitation of DPs causes a significant reduction in the Al concentration in the matrix. The coarse lamellar-shaped DPs are entirely blocked when the aluminium concentration on the matrix is reduced to a very small value [20], and the precipitated phases convert into fine granular or short-lath-shaped CPs. It was also discovered that the DPs and CPs developed in a competitive manner at a medium ageing temperature (200 °C) [19], with the DPs being initiated at grain borders and the CPs being spread throughout the grains. Following T6 (30 h at 200 °C) [19] treatment, a significant amount of β-phases precipitated from the supersaturated solid solution. Typical lamellar-shaped DP colonies began at grain boundaries and spread perpendicular to them. Similar to the T5 sample, several short-lath-shaped CPs grew at front end of such lamellar-shaped DPs. However, in the T6 sample, where the DPs were sparsely dispersed, whole CP areas developed and occupied the recrystallized grain, possibly due to the lower aluminium content being insufficient to induce DP precipitation.

RETRACTED

The microstructure of as-cast AZ80 Mg alloy is effectively changed by adding 1.0% Nd [21]. The grain size of the primary alpha Mg in the alloy diminishes, and its shape shifts from dendritic to the rosette. The coarse eutectic beta Mg phase becomes discontinuous as it refines. In addition, When AZ80 Mg alloys were homogenised at different temperatures, the microstructure revealed a very thin uniform distribution of secondary phases at higher homogenization temperatures compared to lower temperature samples. The secondary phase precipitates as the holding period increases to 6h and 12h, increasing secondary phase precipitation density. At a temperature of 723K [21], the grain size increases as the holding duration increases.

### 3.6 Grain size

Grain size refinement was identified during the reinforcing and extrusion processes. The sizes of grain and texture dispersion of extruded AZ61 barely alter after the post-ageing treatment. The grain size varies depending on the amount of SiCp used, and the number of passes in an equal channel angular pressing operation influences the grain size. The annealing at a higher temperature refinement of grain is the result. The key mechanism for refinement of grain in AZ61 Mg alloy processed at 573 K and 523 K [22]is the formation of twins and the resulting twinning stress, which leads to dynamic recrystallization. As the annealing time and temperature were increased, the size of the ultra-fine grains grew larger [22]. Compared to annealing time, annealing temperature has a large impact on grain development. In AZ91 after the pressure of hydrogen of 7 MPa under 350 °C heat treatment for 24 h, the grain size was decreased to 100–200 nm [3] by hydrogenation disproportionation desorption recombination treatment. Al is also one of the elements that contribute to the HDDR phenomenon, which refines grain size. The amount of Al in the HDDR-treated AZ91 magnesium alloys has little effect on grain size refinement. An inoculated master alloy of Al-3.4V–1B was used for grain structure refinement of the AZ91 magnesium alloy. With 0.6wt% Al-3.4V–1B refiner [23] added, grain size lowered by roughly 60%. The VB2 particles serve as effective nuclei for grain refining in the inoculated alloy of AZ91 with the master alloy of Al-3.4V–1B. In AZ31 when the temperature is below 250 °C, the size of the grain develops slowly. When the temperature of heating exceeds 300 °C [24], the grain size expands dramatically as the temperature rises. In addition, as the holding period is increased, the grain size expands significantly. At 150–250 °C [24] temperature range, the size of the grain grew at first, and then dropped after some time. When the heating temperature exceeds 200 °C, the recrystallization nucleation rate exceeds the rate of growth, resulting in a grain size reduction following recrystallization. In this case, the size of the grain tends to rise as the holding duration at a given temperature increases. The Al–1B-0.6C master alloy has a better grain refining effect on the AZ63 Mg alloy. The grain size of AZ63 Mg alloy can be efficiently reduced from around 170 μm–70 μm by adding 2-wt% Al–1B-0.6C master alloy at 760 °C [25]. It demonstrates the Al–1B-0.6C master alloy's ability to act as a grain refiner. Furthermore, as the alloy temperature rises, the alpha Mg particles in the microstructure coarsen and bond with one another, resulting in smaller grain sizes.

### 3.7 Tensile results of various Mg alloys

In the extruded-rolled AZ31 alloy of magnesium, the heat treatment takes place at various temperatures for varying periods. Extruded rolled alloys have greater strength than as-extruded alloys, while ER alloys have less elongation than as-extruded alloys [26]. The number of twins by the addition of rolling reduction and refines the grain [27], which corresponds to increased strength and decreased flexibility. The orthogonal testing findings reveal that rolling reduction has the greatest impact on tensile strength [28], while the temperature of heat treatment has the greatest impact on elongation. Increased deformation, as a result of adding distortion energy, will make the recrystallization of extruded rolled alloys easier. At 373 K [26], the alloys begin to recrystallize, which is lower than the temperature of recrystallization, when there is enough distortion energy.

RETRACTED

The tensile strength of the AZ31 magnesium alloy, which is under treated by equal channel angular pressing, diminishes as the temperature of annealing rises. That is the specimen's strength, which shows grain size relationships. As the processing temperature rises, the 0.2% proof stress and tensile strength [29] of 2 pass specimens increase. The elongation of the AZ31 alloy under 523 K 2 pass is 25% [29] higher than that of the receiving specimen. As the passes are increased to four under 523 K, the elongation is improved when compared to two passes treated at those temperatures. The tensile properties of 573 K under 4 passes and 2 passes [29], on the other hand, are nearly identical.

Room temperature tensile tests were used to determine the influence of different quenching processes and annealing temperatures on optimum elongation, UTS, and yield strength of coarse-grained AZ61 magnesium alloy. At 350 °C [30], the sample with the optimum elongation was annealed for 2 h before being water quenched. At room temperature, the material's ductility is quite low, with 3.51% [30] of optimum elongation. The AZ61 fine-grain alloy demonstrated greater formability when annealed for 2 h at 350 °C and water quenched, with 5.6% of optimum elongation at failure [30]. The components annealed at 400 °C, which include the UTS, have an average of 258 MPa, which is higher than the components annealed at 350 °C [30], which have a value of 250 MPa. When fine grain samples were compared to coarse grain samples, there was no discernible variation in UTS or yield strength [10]. Elongation increased dramatically at higher forming temperatures, with a maximum elongation of 9.83% [30] for fine grain at 350 °C. Higher forming temperatures obtained a significant decrement in yield strength. At 350 °C temperature of forming, the air quenched sample had the least strength of yield in AZ61 alloy fine grain, with a value of 71 MPa [30]. Water-quenched samples with a yield strength of 161 MPa [30] had the highest strength of yield at 250 °C temperature of forming. At 250 °C, the temperature of forming gave the optimum strength of yield of 139 MPa [30] for the alloy coarse-grained. The strength of tensile was measured at room temperature as well as after heat treatment at 120, 240, and 360 min [8] of soaking time. Furnace heat treatment increased the 0.2% proof strength and UTS of AZ61A magnesium alloy to 313.35 MPa and 217 MPa, respectively [8]. The 0.2% proof strength and UTS were enhanced by extending the period of soaking. The AZ61 magnesium alloys are extruded; they have a superior strength-to-ductility ratio. The tensile strength increases after a further heat treatment at 170 °C of direct ageing treatment for 54 h [12], while the elongation decreases. The technique of extrusion with a high ratio of extrusion improves the AZ61 Mg alloy's ductility and strength, and the direct ageing heat treatment improves both the yield and tensile strengths.

RETRACTED

The stiffness AZ91 treated by cryogenic welding is 206 MPa [31], which is significantly higher than the welded AZ91 without any subsequent treatment. In a cryogenic welding experiment, there appeared to be many Al8Mn5 distributed particles in the heated affection zone [31], which may be responsible for the improved mechanical qualities. The toughness of the sample decreases dramatically when the brittle dendritic phase Mg_17_Al_12_ cracks during the cryogenic process. The emergence of smaller scattered Al8Mn5 and the transformation of dendritic Mg_17_Al_12_ into short rods [31] may be accountable for the material's mechanical qualities. The alloy's strength and elongation rise noticeably following semi-solid squeezing, and even more so after T6 treatment (solution for 24 h at 415 °C + 8 h at 220 °C) [31]. The ultimate tensile strength was achieved a maximum of 285 MPa for squeezing temperature at 575 °C [16] following T6 treatment, while a maximum of 13.36% elongation reached and the strength of elongation of 180 MPa [16] reached which is minimum. T6 treatment enhanced the elongation and UTS of all AZ91 semi-solid compressed alloys of magnesium. On the other hand, all semi-solid alloys' strength of yield is reduced under T6 heat treatment [16]. The elongation and strength of the AZ31 magnesium alloy were both improved by homogenization treatment; the UTS enhanced by nearly 30% and the elongation increased by more than 10% [32]. This is owing to the beta phase refinement and microstructure homogeneity. UTS of the homogenised rolled alloy of AZ91 increases somewhat when compared to the as-rolled specimen, but the elongation increases by nearly 50% [32] in conditions of hot rolling. The stiffness of homogenised rolled improved by roughly 35% [32] after hot rolling, with a little decrease in elongation. This brittle second phase severely limits the enhancement of the ability of forming of AZ91 Mg alloys [33], making subsequent plastic processing more challenging. However, if a tiny crack can be pressed in place using proper rolling technique and the second phase of brittle refined using a heat treatment method, there is enhancement of the properties of mechanical and plasticity [33] of AZ91 alloy of magnesium. As a result, inquiry into the distribution, fragmentation, dissolution and precipitation of the β-Mg_17_Al_12_phase in the AZ91 alloy of magnesium during heat treatment and deformation is critical for enhancing the alloy's strength and plasticity.

RETRACTED

The highest tensile and elongation properties are detected in heat-treated specimens [13]. The reason for this is that this specimen's grain structure is free of precipitations, which means there are no flaws in the alloy's mechanical characteristics. As a result, it has the highest values when compared to the others. It's also been discovered that the ductility and maximum tensile stress of 160 °C [13] aged specimens decline with time. This is attributed to an increase in the content of -precipitate. Similar behaviour was found with 190 °C-aged specimens [13]. Maximum force and elongation are, however, quite minimal in 3-h-aged specimens. Impurities and inclusions in the structure caused by casting flaws may be the cause, and these flaws may impact the structure's mechanical qualities [34]. When the mechanical effects of aged specimens at a temperature of 160 °C and 190 °C were evaluated [13], the aged samples at 190 °C had more maximum stress and deflection than the 160 °C aged samples. For 190 °C aged samples, this could be due to phase precipitations localised in grains rather than grain borders.

The durability (UTS) of the AZ63 Mg alloy improves steadily as the mould temperature rises, while the elongation reaches a greatest value when the temperature reaches 300 °C.But when the temperature increases from 300 °C to 350 °C [14], the elongation reduces slightly. In 350 °C, AZ63 Mg alloy thixo forged exhibits the most complete tensile characteristics. The increase of aluminium solubility in the alpha Mg particles and decrease of the eutectic beta phase has lead to an increase in tensile characteristics in the AZ63 Mg alloy; also, the decrease of the eutectic beta phase is advantageous for enhancing tensile properties. The quantity of MgCO_3_ added to the thixoforged AZ63 alloy boosts both elongation and UTS with the thixoforged alloy with percentage of 1.2 MgCO_3_ having the best tensile properties. Due to increase of temperature of mould from 100 °C to 350 °C [14] the UTS of the thixoforged AZ63 alloy increases. However, when the temperature is attained at 300 °C, the elongation reaches its maximum value. The thixoforged alloy is shown below. These adjustments contributed to the increase of the compactness of the secondary solidified structure and the decrease of the eutectic beta phase due to the fluctuation in solidification behaviour [34], which is dependent on the temperature of mould. Due to this reason, at a time of tensile testing, the crack propagation path will be eventually shifts from along the secondarily solidified structures to completely crossing the α-Mg particles. Reason for this elongation the significant decrease when the temperature approaches 300 °C [14] is the residual local stress concentration caused by partial recrystallization during thixoforging.

RETRACTED

In AZ80 due to grain development and disintegration of β- Mg_17_Al_12_precipitates the strength and elongation of extruded AZ80 alloy specimens after various heat treatments were reduced compared to the extruded AZ80 sample without heat treatment. After solution and ageing treatment, the extruded AZ80 alloy had a better balance of strength and elongation [35]. The resilience of solution treatment and ageing was particularly enhanced at 190 °C [35], which was superior to ageing at other temperatures. The AZ80 sample had the highest strength after H5 treatment (24 h at 190 °C) [35], but elongation was sacrificed. The primary cause was low heat activity, which slowed grain development. In contrast, the formation of CP used to have a precipitation-strengthening impact.

The Nd additive to the AZ80 Mg alloy increases the tensile characteristics in as-cast circumstances when compared to the AZ80 base alloy. When Nd concentration reaches 1.0% [21], the combination properties improve and increase the strength of yield, ultimate tensile strength, and elongation. The characteristics of tensile are compromised by increasing the Nd content from 1.0% to 1.5% [21]. The fine Al_2_Nd and Al_11_Nd_3_ phases, and also the change of the β- Mg_17_Al_12_ phase from continuous to discontinuous precipitate, can improve the tensile properties of the AZ80 Mg alloy. Increasing the Nd concentration, on the other hand, causes the formation of a coarse AlNd stage, which fractures the α-Mg matrix and degrades the mechanical properties. With the addition of 1.0% Nd [21, 36], the yield strength and UTS are enhanced, while the elongation is decreased when compared to as-cast alloys. Fine grains are also good for the tensile characteristics of the AZ80 Mg alloy. The grain size is improved when 1.0% Nd is added, and this refinement improves the alloy's tensile strength. Table 1 shows the summary of pervious research carried out in the AZ Mg alloy.

RETRACTED

**Table 1:** Summary of Mg alloys to improve mechanical properties.

Base material	Process involved	Outcomes	References
AZ61	Inclusion of SiC	SiC particle enhances tensile strength at 1 weight percent but decreases ductility because SiCp is brittle.	Huang et al. [12]
	Hot rolling	In rolled samples microhardness decreases with increase in temperature	Vivek et al. [22]
	Inclusion of Ca	In NaCl solution, the corrosion resistance is improved by the proper Ca content, which is 1% Ca	Chen et al. [37]
	Disintegrated melt deposition method	This dramatically increases compression strength by modifying the grain sizes and basal textures.	Rashad et al. [38]
AZ91	High-Pressure Torsion	In HPT, microstructure gradually changes as torsional strain increases.	Harai et al. [39]
	Equal-channel angular pressing	Grain refinement causes the texture to soften more than it does to strengthen after eight ECAP cycles, increasing yield strength.	Kim et al. [40]
	Friction stir welding	The welded samples may achieve the maximum tensile Strength at a specific rotational speed.	Singh et al. [41]
	Small strain impact forging	As ultimate tensile strength increases, the percentage of elongation steadily decreases because there is a considerable quantity of Mg_17_Al_12_ precipitation.	Jiang et al. [42]
	Friction stir processing	The great strength and ductility of the specimens were mainly due to the widespread dispersion of the texture throughout the crystal.	Luo et al. [43]
	Multi-axial forging	With more multi-axial forging passes, the average grain size shrinks.	Xia et al. [44]
	Multi-directional impact forging	The ductility was increased by 20.6%. Due to the presence of bimodal microstructure.	Jiang et al. [45]
	Hot isostatic pressing	Density and solid solution strengthening are related to ultimate tensile strength.	Liu et al. [46]
	Hot rolling	The as-cast alloy tensile strength is enhanced by hot rolling.	Zheng et al. [32]
	Inclusion of Y_2_O_3_	Mg hybrid nano composites fabricate through microwave shows improvement in microhardness	Ponappa et al. [37]
	Pulse electro deposition	The Ni coating serves as a shield for corrosion	Hajiali Fini et al. [47]
AZ91	Thixoformed	When Si, Sb, Bi, Ca, Sn, and REs react with Mg, the creep resistance increases at high temperatures but has no effect on the creep process.	Roodposhti et al. [48]
	Thixoformed with inclusion of Ca and RE	To improve the creep properties of the AZ91 alloy, Ca and RE elements were added.	Evangelista et al. [49]
	Thixomolding	The process makes the AZ91 Mg alloy less porous and increases its fatigue strength.	Czerwinski et al. [50]
	Inclusion of Si and Sb	In AZ91 + xSi alloys with Sb added, the mechanical characteristics both at low and high temperatures are improved.	Pillai et al. [51]
	Emission of ultrasonic vibration	When increasing ultrasonic power the grain size of the alloy is gradually decreasing.	Gao et al. [52]
	Equal-channel angular pressing	The Mg_17_Al_12_ phase precipitation leads to increase in strength of alloy.	Chen et al. [53]
	Inclusion of Bi and antimony addition	When AZ91 is treated with a trace quantity of bismuth or antimony, it gains yield strength and creep resistance.	Guangyin et al. [54]
	Hydrothermal treatment	As-cast structure of AZ91 becomes more stable and robust due to a decrease in the volume percentage of - Mg_17_Al_12_	Mahmudi et al. [55]
	Squeeze casting	Tensile and hardness parameters in AZ91-2Ca Mg alloy improve with effective mould filling and microstructural refinement.	Goh et al. [56]
	Inoculation and hot deformation	The procedure caused a notable grain refinement as well as the distribution and fracture of intermetallics along the extrusion direction	Mehranpour et al. [57]
AZ31, AZ63	Equal channel angular extrusion	The tensile strength of AZ31 alloy subjected to ECAP falls as the annealing temperature rises.	Yoshida et al. [29]
	High pressure torsion	With an increasing number of HPT turns, the microhardness displays a progressive evolution.	JieXu et al. [7]
	Equal-channel angular pressing	Prior to ECAP processing, initial extrusion reduces grain size, and grain refining becomes more consistent.	Yoshida et al. [29]
	Hydrothermal treatment	Mg alloys demonstrate superior corrosion resistance in simulated concrete pore solutions.	Wang et al. [58]
	Friction stir processing	It demonstrates that this method results in finer and more homogeneous grain structure.	Darras et al. [59]
	Equal channel angular extrusion	After six ECAE passes, the tensile and yield strength values increased by approximately 48% and 87%, respectively.	Mukai et al. [60]
	Thermomechanical processing	Increasing the quantity and size of dynamically recrystallized grains causes the Zener-Hollomon parameter to drop.	Fatemi et al. [61]
	Ultrasonic frequency pulsed arc	Demonstrates an improvement in isotropic tensile strength and good ductility as a result of the equiaxed-grain microstructure.	Cao et al. [62]
	Multi-directional forging with gradient cooling	The grain texture changed as a result of the plastic deformation, increasing the yield strength and tensile strength.	Cui et al. [63]
	Hot rolling	The improvement in microstructure compactness and fine grain strengthening following hot rolling were the key reasons why the alloy's mechanical characteristics improved.	Wang et al. [64]
	Friction stir lap welding	Increase in bonding strength due to the formation of interface microstructure	Fu et al. [65]
	Cold metal transfer process	Due to the varied microstructures in various areas, the tensile characteristics also clearly vary from the deposit's bottom to its top.	Yang et al. [66]
	Wire-arc additive manufacturing	Features lower yield strength, greater elongation, and greater ultimate tensile strength in its anisotropic tensile characteristics.	Wang et al. [67]
	Theorizing	Tensile characteristics are improved by decreasing the eutectic β phase and increasing Al solubility in α Mg particles.	Chen et al. [14]
	Thixoforging	Changes in solidification behaviour, plastic deformation resulted in microstructure evolution.	Chen et al. [14]
	Inclusion of master alloy Al–1B-0.6C	At 760 °C the size of grain reduces after a 2wt% master alloy of Al–1B-0.6C is added.	Guolong Ma et al. [25]
	CeCl3/H2O2 aqueous solution treatment	When the samples are repeatedly immersed in the conversion bath for 30 s–180 s total, better corrosion-resistant surfaces are produced.	Dabala et al. [58]
	Extrusion	After a 10-hour heat treatment at 200 °C, the ultimate tensile strength improved noticeably.	Zhang et al. [68]
	Solid-Liquid Compound Casting	In the transition zone, the hardness steadily increases, lowering interfacial tension and strengthening the interface's bonding capacity.	Dai et al. [65]
	Novel solid-phase processing	The tension-compression asymmetries on the basal texture have been removed, and corrosion resistance and ductility have improved.	Beura et al. [69]
	Friction welding	Tensile strength increases with increasing friction time and friction force.	Anil et al. [70]
	Roll bonding process	When the volume proportion of Mg17Al12 phase decreases, the effect of galvanic corrosion decreases.	Samiei et al. [52]
	Accumulated Roll Bonding	With increased cycles of accumulated roll bonding, the microstructure became finer and grain sizes shrank.	Quang et al. [71]
	Ultrasonic surface rolling	Corrosion resistance is increased when residual compressive stress and nanostructured surfaces are reduced.	Han et al. [72]
	End forming process	With the annealing heat-treatment procedure, formability is increased.	Venugopal et al. [73]
	Inclusion of Sr	Due to the addition of Sr there is positive effects of grain size on the corrosion rate.	Song et al. [74]
AZ80	Inclusion of Nd	Nd addition of 1.0% increases tensile strength	Wang et al. [21]
	Rapid solidification	The corrosion resistance is improved by decreasing grain size.	Aghion et al. [75]
	Equal-channel angular pressing	Under ECAP, the 110∗ die shows a greater grain size than the 90∗ die in AZ80.	Naik et al. [76]
	Chloride solution treatment	In extruded AZ80 magnesium alloy, the cathodic phases provide effective sites for the onset of localised corrosion.	Andreatta et al. [77]
	Differential speed rolling	Increases mechanical strength while significantly reducing formability.	Huang et al. [78]
	Hot multiple forging	The material's mechanical characteristics improve as a result of controlled deformation.	Guo et al. [79]
	Equal channel angular press	After the ECAP procedure, the samples' tensile strength falls, and their compressive yield strength outperforms their tension as the temperature rises.	Wang et al. [80]
	Plasma electrolytic oxidation	Increase in the corrosion resistance in AZ80 Mg alloy.	Pezzato et al. [81]
	Shot peening	On the alloy, a compressive stress layer is detected, as well as increased resistance to corrosion fatigue and cavitation erosion.	Zhang et al. [82]
	High-Pressure Torsion	Superplasticity occurred with a strain rate sensitivity of 0.5, according to microstructural measurements, and the grains were equiaxed after being pulled to the greatest superplastic elongations.	Alsubaie et al. [83]
AZ80	Thermomechanical processing	Extruded nano-composites' hardness increased due to the addition of tougher particles, as well as exceptional grain refinement.	Khosroshahi et al. [84]
	Centrifugal Casting	Due to the presence of more -Mg_17_Al_12_ precipitates, it has been shown that the inner layers have the best mechanical qualities.	Arabi-Nour et al. [85]
	Equal-channel angular pressing	A significant gain in tensile strength,% elongation, and corrosion resistance may be possible depending on the ECAP processing method selected.	Gajanan et al. [76]

RETRACTED

### 3.8 Microhardness results of various Mg alloys

The hardness of AZ61 magnesium alloy was measured at ambient temperature and after heat treatment at different soaking times. After heat treatment, the BHN is reduced as a result of this. BHN is 72.7 before heat treatment and 68 [8] after heat treatment at various holding times. The Brinell hardness number of the Mg AZ61 alloy material is gradually decreasing [8]. The alloy forms coarse granules and a tissue zone of negative [9] in the heat-affected zone during the welding process. As a result, the heat impacted zone in the joint has the lowest hardness value and has the highest value of hardness [9] in the zone of the weld. The discrepancy in β-phase content in the joints was steadily reduced after cryogenic treatment of deep. After the treatment, the microhardness of the heat-affected zone increases the most. The improvement of the sample's overall micro-hardness is dependent on the change in internal stress [11]. Short duration of cryogenic treatment increase the hardness peak [9] appears (4 h). Stress in internal creates a variation that for a short duration, whereas the precipitation of β-phase causes a longer-lasting alteration. The number of particles increases with extended deep cryogenic treatment [9], which plays a key role in enhancing microhardness. When the β-phase precipitation is complete, the second hardness peak appears between 6 and 8 h [9].

The value of microhardness in the rolled AZ61 magnesium alloy falls as the temperature rises. The fall in hardness value is related to the phase present in the AZ61 magnesium alloy and is initially significantly lower [11] in comparison to homogenised and rolled samples. The structure is uniformed through homogenization, whereas the grains in rolled samples are fragmented after rolling, increasing the hardness of AZ61. The principal mechanism for grain refinement in these AZ61 magnesium alloys treated at 523 k and 573 k is dynamic crystallization [22]. When grain refining occurs, the value of microhardness increases, and when the temperature rises, the value of microhardness falls. We can see that when the temperature rises, the sample's hardness diminishes, and that hardness also declines with time in isothermal conditions [22]. The hardness of the metal falls rapidly during the first 60 min of annealing and then stabilises after 120 min [22]. As a result, both temperature and annealing have a substantial impact on the hardness value. The hardness of the fusion sector region is more than that of the heat impacted sector region [31]. The pace of solidification in the laser-weld process is fast, which results in a finer grain structure. The hardness of the weld with a cryogenic treated component is substantially more than that of the welded component in both the heat-affecting sector and the fusion sector [31]. The lattice constant of crystals would drop in cryogenic conditions. From the magnesium base, several Al8Mn5 particles separated. With a Vickers microhardness tester, the hardness of the components was tested to see how treatment of cryogenic affected the microhardness of the AZ91 alloy of magnesium. As a result, the values of microhardness of the FSPed components with cryogenic deep treatment are superior to the FSPed components without cryogenic deep treatment. FSP improves the alloy's microhardness, and deep cryogenic treatment improves it even more. The grain arrangement refinement is thought to be a significant factor in enhancing the AZ91 FSPed alloy hardness. The DCT greatly increased hardness, according to the data. The hardness of AZ91 increased significantly in the squeeze casting of semi-solid, but dropped after T4 (solution for 24 h at 415 °C) [16] treatment, then improved once after T6 treatment, even greater than the as-squeezed. After T6 treatment, the hardness of AZ91 attained its maximum (106.8 HV) at 595 °C squeezing temperature [16]. The hardness of the produced composites increases as the volume% of Y2O3 increases [86]. The addition of hard Y_2_O_3_ particles boosts the load bearing capability of the matrix [86] while also limiting matrix deformation by restricting dislocation migration. Due to heat-treated composites under solution hardening effect have a better hardness than as-casted composite. The reaction of AZ91 composites to heat treatment, increased hardness is greater than that of pure magnesium composites. Intermetallic components and precipitate precipitation are responsible for the enhancement of hardness of the composite of magnesium alloy [87]. The hardness values grew dramatically as the ageing time increased, reaching a maximum value after 24 h, and then decreasing as the ageing period increased. The reduction is due to the effects of ageing. Irrespective of the rate of cooling, the maximum hardness is obtained after 24 h for 20 ° C/s and 0.1 °C/s [87]. The base material microhardness was found to be 56 Hv [4] during the test. In the friction stir processed region, the grain structure was refined and the β-phase was dispersed, which improved the microhardness. The hardness of the specimens aged for 30 min was found to be slightly higher than that of the specimens aged for 60 min [4]. Heat-treated specimens had a higher hardness than the base material, which was 36% higher. At a temperature of 200 °C, these components were aged for 30 min and 60 min [4], respectively. At 200 °C temperature for ageing, the fineness of grain is comparatively good. The hardness of the specimens changes along their transverse section. The hardness of the base material zone was low, but it began to rise in the thermomechanically affected zone and reached a peak in the nugget zone [28]. The grains coarsen up to 25.5 μm of the average size of grain after being annealed at 773K for 4 h [29], with a significant decrement in hardness as a result of abnormal growth of grain. As the number of high-pressure torsion turns increases, the microhardness homogeneity of AZ31 Mg alloys processed by HPT shows a gradual evolution. It shows an evolution towards a homogeneous distribution after ten HPT turns, i.e., hardness homogeneity across HPT discs is achieved after ten turns with a saturation hardness value of 125 [7]. Because of its larger grain size, smaller twin fraction, and lower dislocation density, the as-homogenized sample has the lowest microhardness [27]. The microhardness dispersion along with thickness for the as-homogenized sample, on the other hand, is not uniform. That is, it has the highest value of microhardness fluctuation. Because the size of grain decreased [28] and the twin% and density of the shear band increased when the thickness was reduced, the average microhardness increased.

RETRACTED

According to the findings of microhardness tests, the result of the as-cast AZ63 alloy will decrease after solution heat treatment. It is found to be that the microhardness of the as-cast AZ63 specimen is 70.5 HV [13]. The microhardness of the specimens drops to around 63 HV [13] after air cooling following the solution heat treatment. At a temperature of 160 °C, the microhardness fluctuates very slightly throughout the ageing process. The maximum microhardness value was 71.1 HV after 9 h of ageing [13], and the minimum microhardness value was 63.7 HV after 6 h of ageing. The microhardness of AZ63 Mg alloy does not appear to be affected by ageing at 160 degrees Celsius [13]. Before the ageing at 190 °C, microhardness does not change, but after more than 3 h of ageing, a very straight increase in microhardness can be detected. The specimen's microhardness begins to increase significantly after 6 h of ageing. As a result, more than 6-h of ageing at 190 °C [13] required to improve the microhardness of AZ63 Mg alloy.

According to the findings of microhardness tests, the result of the as-cast AZ63 alloy will decrease after solution heat treatment. It is found to be that the microhardness of the as-cast AZ63 specimen is 70.5 HV [13]. The microhardness of the specimens drops to around 63 HV [13] after air cooling following the solution heat treatment. At a temperature of 160 °C, the microhardness fluctuates very slightly throughout the ageing process. The maximum microhardness value was 71.1 HV after 9 h of ageing [13], and the minimum microhardness value was 63.7 HV after 6 h of ageing. The microhardness of AZ63 Mg alloy does not appear to be affected by ageing at 160 degrees Celsius [13]. Before the ageing at 190 °C, microhardness does not change, but after more than 3 h of ageing, a very straight increase in microhardness can be detected. The specimen's microhardness begins to increase significantly after 6 h of ageing. As a result, more than 6-h of ageing at 190 °C [13] required improving the microhardness of AZ63 Mg alloy.

The as-extruded material (69.1 Hv) exhibited higher initial hardness than the T4 material (66.6 Hv) because of the finer grains and precipitates present [19]. The ageing time necessary to achieve maximum hardness, or apex time, for the as-extruded alloy was 15 h, which was half the time required for the T4 material (30 h) [19]. The hardness increment per hour from the unaged to the apex condition of the as-extruded material was 1.68 HV, which was significantly higher than the T4 material's (0.88 Hv) [19]. The as-extruded material's higher dislocation density facilitates the nucleation and growth of precipitates [20] by providing diffusion channels for alloying atoms, resulting in a faster age-hardening tendency.

RETRACTED

At higher homogenization temperatures of 623 K and 723 K [88], the alloy's average micro hardness value was dramatically reduced. This is due to the partial relaxation of internal tensions that occurs during the healing and grain growth process. The alloy's hardness rose when the holding period was increased due to considerable diffusion of secondary phases in the Mg matrix [20], which boosted the alloy's hardness. After homogenization at temperatures above 573 K [88], the average microhardness decreases slightly. However, increased holding times resulted in better microhardness due to secondary beta phase dispersion along grain boundaries, and the alloy's hardness rises as grain size decreases.

### 3.9 Corrosion behaviour of AZ series Mg alloy

In Mg–Al based alloy the phase of β serves as a barrier to corrosion and a cathode. The phase of α has an impact on the alloy's corrosion rate. The α-phase can be refined to cause the continuous network of formation of the phase of β around the phase of α [9] and thereby resistance to corrosion of magnesium alloys enhanced. A continuous network of the phase of β is scattered throughout the matrix of α after substantial treatment of cryogenic, and the refined β-phase can improve the α-matrix's organisation. The β-phase is also vital in preventing the α-phase from peeling away from the surface. The β-phase is far more difficult to work with than the phase of α. Chemical inertia is likewise high in the β-phase. When the β-phase content is low, the α-phase is more easily eroded [9]. Nonetheless, the β-phase's high potential is beneficial to corrosion resistance. In general, the β-phase actively contributes to the corrosion resistance of the joints. They were in the NaCl solution immersed for 10 h [9] without the deep cryogenic treatment. The dispersed network of β-phase in the joint of weld prevents corrosion from spreading further. The source of corrosion is the same across the joint, however, the corrosion resistance varies. Following various periods of treatment of cryogenic deep, the components were submerged in NaCl solution for 20 h [9]. The damage of corrosion on the surface of the component grows as the deep cryogenic treatment period decreases, and most pits emerge on the α-phase surface. When the cryogenic treatment period is 8 h [9] some pits of inlay of white are there, the white material is the corrosion product, and it is spread on the α phase surface oddly. The pits have 15.33 m [9] of optimum diameter. When the treatment of cryogenic deep duration is 6 h, microscopic cracks emerge all over the pits that progressively spread outward, and the metallic sheen of the components steadily fades. When the treatment of cryogenic deep period is 6 h, the component surface corrodes [9]. Microstructural variations have a significant impact on the corrosion behaviour of AZ61 magnesium alloy welded joints. The deep cryogenic treatment causes microstructural changes in the joints, that help to enhance the corrosion resistance of the joint. In NaCl solution, this alloy shows severe corrosion, with corrosion rates of 3.46 and 4.96 mm/a at 3.5% [89] and 0.5% NaCl solution. The corrosion behaviour of the alloy reduces at first, then significantly rises with the addition of Ca. When the concentration of Ca is 1%, there is the lowest rate of corrosion of AZ61 magnesium alloy [89]. When the content of Ca is increased to 2% [40], the corrosion rate increases significantly. In 0.5% NaCl solution the rate of corrosion is always lesser than those in 3.5% NaCl solution [89], indicating that the concentration of NaCl solution has a greater impact on the behaviour of corrosion of AZ61 alloy of magnesium. The resistance to corrosion of AZ61 alloy of magnesium in NaCl solution can be increased by adding the right amount of calcium. The corrosion surface of AZ61 with 1% Ca magnesium alloy [90] is exceptionally homogenous and dense, which is why the corrosion rate is so low. The major components of this alloy are α-Mg, Al_8_Mn_5_, and Mg_17_Al_12_. In the Al_8_Mn_5_ phase, the Fe particles are separated. With reducing impurity element Fe concentration in the solution treatment, cast, and ageing circumstances, the rate of corrosion and area of the alloy of AZ61 decreased. The lowest corrosion rate is achieved with solution treatment.

RETRACTED

According to the findings, the rate of corrosion of FSPed components with cryogenic treatment was enhanced in comparison to components without cryogenic treatment. When compared to the corrosion rate as as-received with cryogenic treatment and without cryogenic treatment, the value of the corrosion rate 0.080663 mm/year [15] was best at processing settings of 1250 rpm and 30 mm/min [15] with cryogenic treatment. The corrosion rate increased when the tool rotation speed and tool traverse speed increased, compared to previous values. Without cryogenic treatment, the corrosion rate of the as-received alloy was 0.300469613 mm/year [15] after cryogenic treatment, it was 0.248711 mm/year.

The rate of corrosion for all specimens in semisolid squeezing is different and depends on the heat treatment environment. In comparison to as-cast, T4 has a high corrosion rate [90]. T6-12 h specimens have the lowest corrosion rates among T6. T6-22 h, on the other hand, showed a higher rate of corrosion over time [90] due to a micro fracture on the surface specimen, which was corroded easily. Two elements influence the rate of corrosion generated by heat treatment. First, due to precipitates of β around grain boundaries, the rate of corrosion decreases. The second factor is the increased rate of corrosion caused by the α-matrix's lower aluminium concentration. T4 has a higher rate of corrosion across the entire surface. Although there was a lot of aluminium in the α-Mg phase during T4, the natural protective film oxide layer was quickly broken down due to weak localised residual phase sites. When compared to other metrics, T6-12 h has a reduced rate of corrosion during ageing [90]. Because of an imbalance in the phase precipitates distribution as well as the aluminium concentration in the α-Mg matrix, the rate of corrosion was higher after T6-12 h than before T6-12 h.

The use of a Ni coating improves corrosion resistance. The Ni coating functions as a shield against corrosion, preventing corrosion of the substrate [91]. The addition of nanoparticles of Sic to the coating improves corrosion resistance even further. It lowers the coating's submicron flaws and prevents corrosive media from reaching the coating's surface. Ceramic particles such as WC, Al_2_O_3_ and Sic have excellent corrosion characteristics, and their inclusion in the coating enhances corrosion resistance. In the present study, adding Ti to AZ91 alloy may reduce the corrosion rate and current, with AZ91-0.8Ti alloy having the lowest rate of corrosion value and AZ91-0.4Ti alloy having the lowest corrosion current density [18]. Grain refinement and beta phase changes to small uniformly distributed beta phases are the main reasons for the enhanced resistance to corrosion of the AZ91-Ti alloy.

The corrosion mechanism of the base material, FSP specimen, and heat-treated specimens was investigated using an immersion corrosion test. After 24 h of immersion, the corrosion rate of the base material was 2.52 mm/year [4], while that of the FSP specimen was 2.08 mm/year [4] (20% less). Following 48 h of immersion, the least corrosion rate after heat treatment is recorded, which is 2.18 mm/year (15% less) [4]. The base material had a corrosion rate of 2.99 mm/year, the FSP specimen had a rate of 2.15 mm/year (38% less), and the heat-treated specimen had a rate of 1.76 mm/year (69% lesser) [4]. In comparison, after 48 h of immersion in heat-treated specimens, the corrosion rate steadily decreases. This is due to the creation of a corrosion layer, which slowed the pace of deterioration. Furthermore, the boundary of grain served as a protection against corrosion activity, slowing the rate of corrosion in heat-treated specimens. For heat-treated specimens, the rate of corrosion of heat-treated specimens appears to be lower than that of the base material [5]. The drop-in corrosion rate is due to the phase's fine dispersion and an increase in the grain boundary, which resulted in a reduction in corrosion activity. As a result of the FSP and heat treatment process, the corrosion resistance was enhanced.

RETRACTED

The resistance to corrosion of this Mg alloy is greater in saturated Ca(OH)_2_ than in Ca(OH)2 diluted with 3.5wt% NaCl solution [92]. In both types of test solutions, corrosion resistance improves dramatically after hydrothermal treatment. The corrosion resistance of AZ31 alloy coated with simulated concrete pore solution improved in both the Cl- and non-Cl-solutions [92]. Due to the alkalinity of the solutions, Mg alloys demonstrate superior corrosion resistance in simulated concrete pore solutions. The corrosion behaviour of magnesium alloy is altered when chloride ions are added to simulated concrete pore solutions. The corrosion resistance after hydrothermal treatment is also increased in simulated concrete pore solution with and without the addition of chloride ions [92] due to the compact microstructure of the hydrothermal coating.

The grain size has a significant impact on the corrosion behaviour of an alloy. The stable passive oxide layers block the grain boundary during the process [57], making it a non-relatively active site in comparison to the grain. The implementation of the accumulative roll bonding technique results in a considerable reduction in grain size. By increasing the number of process cycles, the corrosion resistance is enhanced [57]. Fine-grain transports more detached oxide layers, which act as an erosion boundary. Because of its moo division and separated dispersion, the Mg_17_Al_12_ stage functions primarily as a micro-galvanic cathode to accelerate erosion. Because the volume rate of Mg_17_Al_12_ stage decreases after ARB preparation, the galvanic erosion effect is reduced. After 24 h in seawater, the corrosion products of the AZ63 Mg alloy samples primarily consisted of CaCO_3_ and Mg(OH_)2_, whereas the corrosion products after 24 h in a 3.5 wt.% NaCl solution [46] primarily consisted of Mg(OH)_2_ and Mg_2_(OH)_3_Cl_4_H_2_O. The corrosion potential of the seawater samples was lower than that of the 3.5 wt.% NaCl solution samples, and the corrosion current density was also lower in the seawater samples than in the 3.5 wt.% NaCl solution samples. The Mg alloy AZ63 corrodes more slowly in seawater than in a 3.5 wt.%NaCl solution, according to the findings [46]. The corrosion resistance of the AZ63 Mg alloy immersed in natural saltwater was superior to that of the former due to the compact deposits that grew on the former. After four runs of ECAP, this process through die at 598 K [76] results in a decreased corrosion rate. The reduced derangement density at the temperature of recrystallization is the fundamental reason for this. As a result of the reduced particle size and increased secondary phase dispersion, corrosion resistance improves. The corrosion resistance of the AZ80 Mg alloy was also increased by rapid solidification [76].

RETRACTED

## 4 Conclusions

The effect of heat and cryogenic treatment on the mechanical and corrosion properties of AZ series Mg alloys has been demonstrated in this review of various magnesium alloys. Based on processes under various temperature conditions, there were changes in microstructure and also grain refinement. Grain refinement improves mechanical behaviour and hardness of the magnesium alloy. However, it reduced the corrosion resistance properties. The majority of the research work has been carried out using AZ series Mg alloys. It is expected that the effect of heat and cryogenic treatment on other Mg alloys will be studied in the future.

## Declarations

### Author contribution statement

All authors listed have significantly contributed to the development and the writing of this article.

### Funding statement

This research did not receive any specific grant from funding agencies in the public, commercial, or not-for-profit sectors.

### Data availability statement

No data was used for the research described in the article.

### Declaration of interest’s statement

The authors declare no conflict of interest.

### Additional information

No additional information is available for this paper.
